This article has been retracted.

# M2 macrophage-derived extracellular vesicles promote gastric cancer progression via a microRNA-130b-3p/MLL3/GRHL2 signaling cascade

**DOI:** 10.1186/s13046-020-01626-7

**Published:** 2020-07-13

**Authors:** Yu Zhang, Wenbo Meng, Ping Yue, Xun Li

**Affiliations:** 1 The First Clinical Medical School of Lanzhou University, Lanzhou, 730000 Gansu Province People’s Republic of China; 2 Department of Thoracic Surgery, The First Hospital of Lanzhou University, Lanzhou, 730000 People’s Republic of China; 3 Department of Special Minimally Invasive Surgery, The First Hospital of Lanzhou University, Lanzhou, 730000 People’s Republic of China; 4 Department of General Surgery, The First Hospital of Lanzhou University, No. 1, Donggang West Road, Chengguan District, Lanzhou, 730000 Gansu Province People’s Republic of China

**Keywords:** Gastric cancer, microRNA-130b-3p, M2 macrophages, Extracellular vesicles, MLL3, GRHL2

## Abstract

**Background:**

Transfer of noncoding microRNAs (miRNAs) by extracellular vesicles (EVs) promotes the development of chemoresistance in many tumor types. Additionally, restoration or depletion of several miRNAs has been observed in multiple cancer types including gastric cancer (GC). In this present study, we aimed to investigate the mechanism of miR-130b-3p in M2 macrophage-derived EVs in the development of GC through regulation of mixed lineage leukemia 3 (MLL3) and grainyhead-like 2 (GRHL2).

**Methods:**

Expression of miR-130b-3p and GRHL2 was quantified in 63 pairs of cancerous and noncancerous gastric tissues. The predicted binding between miR-130b-3p and MLL3, together with the enrichment of MLL3, H3K4me1, and H3K27ac in gene enhancer region, was verified by luciferase activity assay and chromatin immunoprecipitation. Effects of miR-130b-3p on GC cell proliferation, apoptosis, migration and invasion, as well as tube formation of human umbilical endothelial vein cells (HUEVCs) were further determined by gain- and loss-of function assays in vitro.

**Results:**

miR-130b-3p was upregulated in GC tissues, and miR-130b-3p promoted survival, metastasis and angiogenesis of GC cells as well as enhanced tumor formation and angiogenesis in GC in vivo. Additionally, miR-130b-3p delivered in M2 macrophage-derived EVs promoted survival, migration, invasion, and angiogenesis of GC cells. Notably, MLL3 inhibited GC cell proliferation, migration, invasion, and vessel-like tube formation of HUEVCs by increasing GRHL2. Furthermore, downregulation of miR-130b-3p in M2 macrophage-derived EVs or upregulation of GRHL2 inhibited tumor formation and angiogenesis in GC.

**Conclusion:**

This study highlights that EVs loaded with the specific miRNA cargo miR-130b-3p mediate communication between M2 macrophages and cancer cells in the tumor microenvironment through the modulation of MLL3 and GRHL2 in GC.

## Background

Gastric cancer (GC) is the fourth most prevalent cancer and second leading cause of cancer-associated mortality across the world [1]. About 50% of GC incidence occurs in East Asian countries, which also exhibit a higher death rate from this disease compared to other countries [2]. The risk factors for GC include *H. pylori* infection, obesity, smoking, alcohol, salt intake, fiber intake, as well as family history of GC [3]. Apart from regular systemic imaging, endoscopic examination, and locoregional imaging, the detection of GC-associated biomarkers, along with circulating tumor cells are of great importance to the timely diagnosis of GC [4]. Although surgery is the most useful and effective treatment for localized GC, about 50% of patients with advanced GC experience recurrence after initially curative resection [5]. Furthermore, the prognosis remains poor for patients with recurrent or unresectable advanced GC, who have less than 12 months median survival time with conventional therapy [1]. Thus, with the ultimate aim to reduce the socioeconomic burden associated with GC, it is essential to identify novel biomarkers for GC therapy.

Macrophages are the main population of tumor-infiltrating immune cells, and M2 macrophages can induce tumor progression by enhancing tumor angiogenesis and metastasis [6]. Numerous types of cells are able to release extracellular vesicles (EVs), and their transmission can regulate therapeutic resistance of cancer cells embedded among tumor microenvironment cells [7–9]. A recent study has underlined the potential role of EVs in GC diagnosis and management [10], while other research indicates that M2 macrophage-derived EVs induce the migration of GC cells [11]. Non-coding microRNAs (miRNAs) are dis-regulated in GC, which implicates their involvement in GC development and progression [12]. Previous studies have shown that miR-130 plays a cancer-promoting role in tumors [13–15], and that it promotes the proliferation and migration of GC cells by binding to transforming growth factor beta receptor II [16]. Mixed lineage leukemia 3 (MLL3), located on chromosome 7q36.1., a member of the TRX/MLL gene family, is regarded as a vital poor prognostic factor for GC [17]. Expression of MLL3 in GC may be involved in patient survival after curative resection, implying that MLL3 is an independent biomarker for disease recurrence [18]. MLL3 can regulate H3K4me1 and thus mediate gene enhancer activity [19, 20], and other research shows that it binds to the target gene grainyhead-like 2 (GRHL2) enhancer region H3K4me1 to promote the expression of GRHL2 [21]. Based on these lines of evidence, we speculate that miR-130b-3p in M2 macrophage-derived EVs could regulate GRHL2 through MLL3, and thus promote the development of GC.

## Materials and methods

### Ethics statement

All animal experiments were conducted in compliance with the Guide for the Care and Use of Laboratory Animal by International Committees. Patients gave informed, written consent for tissue donation. The protocol was approved by the Institutional Animal Care Use Committee of the First Hospital of Lanzhou University, the First School of Clinical Medicine.

### Human tissue specimen and human GC cell lines

Sixty-three pairs of paraffin-embedded cancerous and adjacent noncancerous gastric tissues were provided by the First Hospital of Lanzhou University, the First School of Clinical Medicine. GC cell lines (NUGC-3, HGC27, MKN45, AGS), human normal gastric mucosal cells (GES-1), human umbilical endothelial vein cells (HUEVCs), and human mononuclear macrophage cell lines (THP-1) were purchased from the American Type Culture Collection (ATCC, https://www.atcc.org/). The complete medium was at centrifuged at 100,000×g at 4 °C overnight to remove EVs [22]. GC cell lines and HUEVCs were cultured in Dulbecco’s Modified Eagle’s medium (DMEM) (31600–034, Hyclone, Logan, UT, USA) containing 10% fetal bovine serum (FBS, 10099141, Gibco, Grand Island, NY, USA). THP-1 cells were cultured in Roswell Park Memorial Institute-1640 medium containing 10% FBS. All the cells were incubated in an incubator at 37 °C with 5% CO_2_ under saturated humidity. When reaching 90% confluence, cells were passaged at 1:3–1:4. The cell lines were all verified by STR analysis and were free of mycoplasma contamination [23]. THP-1 cells were treated with 100 ng/mL polarized 12-myristate 13-acetate (P8139, Sigma-Aldrich, St. Louis, USA) for 24 h for differentiation into macrophages, and with 20 ng/mL interleukin-4 (IL-4) (AF-200-04-5, Peprotech, NJ, USA) for 72 h for differentiation into M2 macrophages.

### Fluorescence in situ hybridization (FISH) and immunofluorescence

A two-step immunofluorescence process was adopted for ISH assay. Firstly, FISH was performed using Locked Nucleic Acid technology developed by Exiqon (Copenhagen, Denmark) to realize the superior hybridization property for detection of miR-130b-3p in situ. To further improve detection sensitivity, double-digoxigenin (DIG)-labeled probes (hsa-miR-130b-3p, 610,948–360, Exiqon) were introduced. The results were visualized by means of Tyramide Signal Amplification (TSA) Plus Fluorescein System, an upgraded version of standard tyramide system, TSA Plus Fluorescein System (NEL741B001KT, Perkin Elmer, Waltham, MA, USA). Secondly, immunofluorescence was conducted using antibody to CD206 (sb64693, Abcam Inc., Cambridge, MA, USA). In the FISH assay, sheep antibody to DIG-peroxidase (11,207,733,910, Roche Life Science, Basel, Switzerland) was used before incubation with TSA. The secondary antibody for fluorescence detection was Alexa Fluor® goat-anti-rabbit (568) (A-11011, Thermo Fisher Scientific, Invitrogen, Carlsbad, CA, USA). SlowFade®Gold anti-fade reagent containing 4′,6-diamidino-2-phenylindole (DAPI) (S36938, Life Technologies, Carlsbad, CA, USA) was used as the mounting medium. Double-DIG-labeled U6 small nuclear RNA (U6, hsa/mmu/rno, 699,002–360, Exiqon) and Scramble-miR (699004–360, Exiqon) probes served as positive and negative controls (NCs), respectively.

### Cell transfection or lentivirus infection

When M2 macrophages in the logarithmic growth phase had reached 30% confluence, they were infected with lentivirus with miR-130b-3p overexpression or knockdown. About 2 × 10^6^ TU of corresponding lentivirus and 5 μg of Poly-brene were added to 1 mL serum-free and antibacterial medium, and the cell transfection was observed under an inverted fluorescence microscope (IX71, Olympus, Tokyo, Japan) for 2–3 d. After transfection for 48 h, 1 μg/mL of puromycin was added to each well to screen out the stably transfected cells, and the cells were cultured for several days to obtain the stably transfected cells, which were then further cultured in conventional medium. MLL3 overexpressing or knockdown lentivirus, GRHL2 overexpressing lentivirus and its NC were used to infect NUGC-3 and HGC27 cells in the same manner. Lentiviruses were all purchased from Invitrogen. miR-130b-3p agomir or miR-130b-3p antagomir and its corresponding NC (Creative Biogene, NY, USA) (final concentration: 100 pmol) were introduced into NUGC-3 and HGC27 cells using lipofectamine 2000 reagent according to the manufacturer’s instructions (Invitrogen). NUGC-3 and HGC27 cells were also treated with M2 macrophage-derived EVs or M2 macrophage-derived EVs with knockdown of miR-130-3p or M2 macrophage-derived EVs with overexpression of miR-130-3p or M2 macrophage-derived EVs with overexpression of miR-130-3p and overexpression of GRHL2.

### EV isolation and identification

When the M2 macrophages reached 80–90% confluence, the complete medium was discarded, and 30 mL of cell culture medium was collected from each cell line. EVs were isolated by differential centrifugation as previously described [22]. EVs were isolated according to the instructions of ExoQuick (System Bioscience, Mountain View, CA, USA). The pellet after centrifugation was resuspended and stored at − 80 °C until use.

EVs were identified by examination under a transmission electron microscope. The sample was adsorbed onto a carbon-coated nickel grid and stained with 2% methylaminotungstate for 5 min. The excess stain was then wiped from the grid with filter paper and the grid was washed twice with distilled water, followed by drying. Then, the sample was inspected at an acceleration voltage of 80 kV in a JEM-1230 electron microscope (Nihon Denshi, Tokyo, Japan). Particle size analysis of EVs was performed using nanoparticle tracking analysis (NS300, Malvern Instruments Co., Ltd., Worcestershire, UK) [24]. Western blot analysis was used to identify the surface markers of EVs. After the suspension of EVs was concentrated, the protein content was determined by bicinchoninic acid kit (23,227, Thermo Fisher Scientific). Sodium dodecyl sulfate polyacrylamide gel electrophoresis was undertaken, followed by protein denaturation and electrophoresis, and the protein was transferred onto the membrane. The expression of specific marker proteins of EVs, such as tumor susceptibility gene 101 (TSG101), CD63 and CD81, was determined by quantitative western blotting.

### Labeling and tracking of EVs

The EVs (20 μg) were labeled with PKH67 Green Fluorescent membrane linker dye (Sigma-Aldrich) according to the manufacturer’s instructions. The labeled EVs were then resuspended and added to unstained NUGC-3, HGC27 and HUEVCs for uptake of EVs. After incubation at 37 °C for 12 h, the uptake of EVs by cells was observed under a confocal microscope (Zeiss Meta 510, Thornwood, NY, USA).

### Reverse transcription quantitative polymerase chain reaction (RT-qPCR)

TRIzol reagent (Invitrogen) was used to extract total RNA according to the manufacturer’s instructions. RT was performed using a PrimeScript RT reagent Kit (Promega, Madison, WI, USA). After that, gene expression was quantified using SYBR Green Master Mix (Life Technologies). Total RNA extraction was performed using the miRNeasy Mini Kit (217,004, QIAGEN, Hilden, Germany). RT of miRNA and following qPCR were performed using miScript II RT kit (218,161, QIAGEN) and miScript SYBR® green PCR kit (218,075, QIAGEN). Primer sequences are synthesized by Invitrogen (Table 1). Real-time qPCR was performed using an ABI 7500 qPCR apparatus (Applied Biosystems, Life Technologies, CA, USA). U6 was a loading control for miR-130b-3p, and glyceraldehyde phosphate dehydrogenase (GAPDH) served as an internal reference of other genes. 2^-ΔΔCt^ was used for calculating the expression of genes.

**Table 1:** Primer sequence for reverse transcription quantitative polymerase chain reaction

Gene	Sequence (5′-3′)
miR-130b-3p	F: 5′-TTCACATTGTGCTACTGTCTGC-3’
	R: 5′-GCTCTGACTTTATTGCACTACT-3’
MLL3	F: 5′-TGCCTGTTCTCAGTGTGGTC-3’
	R: 5′-TCACACAGCAGGAGTCTTCC-3’
GRHL2	F: 5′-AACAGGAAGAAAGGGAAAGGCCAGG-3’
	R: 5′-TAGATTTCCATGAGCGTGACCTTG-3’
U6	F: 5′-CTCGCTTCGGCAGCACA − 3’
	R: 5′-AACGCTTCACGAATTTGCGT − 3′
GAPDH	F: 5′-GTCTCCTCTGACTTCAACAGCG − 3’
	R: 5′-ACCACCCTGTTGCTGTAGCCAA − 3′

*F* forward, *R* reverse, *miR-130b-3p* microRNA-130b-3p, *MLL3* mixed lineage leukemia 3, *GRHL2* grainyhead-like 2, *GAPDH* glyceraldehyde phosphate dehydrogenase

### Western blot analysis

The total protein was extracted by radioimmunoprecipitation assay buffer (Sigma), with the concentration measured by a bicinchoninic acid assay kit. The extracted proteins were separated and then transferred onto nitrocellulose membranes (Millipore, Bedford, MA, USA). Next, the membranes were blocked with 5% bovine serum albumin for 1 h, and then added with primary antibodies to B-cell lymphoma-2 (Bcl-2) associated protein X (Bax) (ab182733, 1:1000), Bcl-2 (ab32124, 1:1000), cleaved caspase 3 (ab2302, 1:1000), total caspase 3 (ab13847, 1:500), GAPDH (ab181602, 1:10,000) (all from Abcam), and vascular endothelial growth factor (VEGF, sc-4570, 1:1000, SANTA CRUZ, Japan) and incubated at 4 °C overnight. On the next day, the membrane was then incubated with relative secondary antibody, goat anti-rabbit polyclonal immunoglobulin G (IgG) antibody diluted with 5% skim milk (ab205718, 1:5000, Abcam), and developed by chemiluminescence reagent and Gel imaging system (Bio-Rad, USA). Quantitative analysis was performed using IPP7.0 software (Media Cybernetics Inc., Rockville, MD, Singapore).

### Luciferase activity assays

HEK293T cells (ATCC) were cultured in an incubator at 37 °C with 5% CO_2_ and saturated humidity, and DMEM (Sigma-Aldrich) was renewed once every 2 or 3 days. The HEK293T cells were co-transfected with wild-type (WT) or mutant type (MUT) MLL3 3′-untranslated region (3′-UTR) psiCHECK-2 plasmid (Promega) and miR-130b-3p/mimic or mimic NC using lipofectamine 2000 (Invitrogen). Cell lysates were collected 48 h post transfection and then firefly and renilla luciferase activities were measured by a dual luciferase reporter assay kit (Promega) based on the manufacturer’s protocol. Renilla luciferase activity was utilized for normalization.

### Chromatin immunoprecipitation (ChIP) assay

The cell lysate was sonicated and then MLL3 antibody, H3K27ac (ab4729, 2 μg for 25 μg of chromatin, Abcam), H3K4me1 (ab8895, 2 μg for 25 μg of chromatin) antibody or non-specific IgG (ab171870, 1:1000, Abcam) for immunoprecipitation. After multiple washes, immunoprecipitated DNA was used for RT-qPCR to detect GRHL2 expression. Anti-MLL3 (for ChIP) was generated against the aa 2951–3091 (α-MLL3-MR) or aa 443–590 (α-MLL3-NTD) of MLL3 protein in house.

### Cell counting kit-8 (CCK-8) assay

The experimental procedures were carried out according to the Dojindo Cell Counting Kit-8 (Kumamoto, Japan). Here, 2 × 10^3^ cells were seeded into 96-well plates per well and then cultured for 24 h. CCK-8 reagent (10 μL) was added into 100 μL complete medium, and incubation continued in the cell culture incubator. The absorbance value at 450 nm (Multiskan FC microplate reader, 51,119,100, Thermo Fisher Scientific) was detected at different time points (0, 24, 36, 48, and 72 h).

### Terminal dexynucleotidyl transferase (TdT)-mediated 2′-deoxyuridine 5′-triphosphate (dUTP) nick end labeling (TUNEL) staining

The apoptosis-positive cells of brain tissues of each group were detected according to the DeadEnd™ fluorescent-labeled TUNEL detection kit (Promega). Under a laser confocal microscope (Nikon, Tokyo, Japan), the nuclei were stained blue by DAPI, and the apoptosis-positive cells were stained green. Five high-power fields (× 400) were randomly selected from each group, and the number of apoptotic cells was counted by inputting the ImageProPlus image analysis processing system (Motic Med 6.0 system, USA). Apoptotic cell rate = number of green apoptotic cells/number of blue cells × 100%.

### Transwell assay

Matrigel (EMD Millipore, Merck KGaA) was equilibrated overnight to a liquid state, and 200 μL Matrigel was supplemented with 200 μL serum-free medium, and then mixed well to dilute Matrigel. Next, 50 μL Matrigel was added to each Transwell plate, and incubated for 2–3 h to insure a solid state. A cell suspension was prepared using medium containing 20% FBS, 200 μL cell suspension was added to the apical chamber of each well, and 800 μL conditioned medium containing 20% FBS was added to the basolateral chamber. The transwell plate was then rinsed with formaldehyde for 10 min, washed three times with water, and stained with 0.1% crystal violet staining solution. The cells on the upper surface were wiped away with cotton balls, and the Transwell bottom chamber was observed under an inverted microscope (IX71, Olympus). Transwell migration experiments did not require Matrigel coating, and the incubation period was 16 h. Cells from at least four randomly-selected visual fields were counted.

### Matrigel-based angiogenic assays

Matrigel (EMD Millipore, Merck KGaA) were placed in a refrigerator at 4 °C overnight to melt into a yellow gel-like liquid. The yellow gelatinous liquid (10 μL) with the thickness of 0.5 mm was taken up in a glass pipette and applied to the pre-chilled angiogenic slides (81,506, ibidi, Munchen, Germany). After 24 h, HUEVCs were harvested and resuspended in DMEM to make a cell suspension after 1 h of starvation without serum. The cell suspension (50 μL) with a density of 2 × 10^5^ cells/mL was seeded into the Matrigel-coated slides, and the cell culture medium of the corresponding group was supplemented to each well, with three replicate wells set for each group. After 12 h, photographs were taken under a Leica inverted phase contrast microscope (× 100). The number of complete capillary lumens surrounded by cells was calculated by Image-Pro Plus (version 6.0) in at least three fields in each group.

### Tumor xenograft in nude mice

Fifty male BALB/c nude mice raised at the Animal Experiment Center of Lanzhou University, (Lanzhou, Gansu, China) following good laboratory practice aged (5–7) weeks and weighing (18–22) g were selected for the study. miR-130b-3p agomir, miR-130b-3p antagomir, M2 macrophage-derived EVs, M2 macrophage-derived EVs with knockdown of miR-130-3p or overexpression of GRHL2 that had been transfected into NUGC-3 and HGC27 cells were injected into the tail vein of nude mice. NUGC-3 and HGC27 cells in logarithmic growth phase were collected, and the cell suspension concentration was adjusted to 1 × 10^6^ cells/100 μL with PBS. The 100 μL cell suspension was injected subcutaneously into the right groin of the mice, and M2 macrophage-derived EVs or normal saline was injected into through the caudal vein. After 28 days, nude mice were euthanized by CO_2_, tumor tissues were dissected, and tumor masses were measured and photographed. Subsequently, the tumor mass was stored in liquid nitrogen. The remaining tumor mass and other organs were immersed in 4% paraformaldehyde overnight and processed by wax embedding for immunohistochemistry analysis. Tumor volume (V) = [length (L) × width (W)]^2^/2.

### Immunohistochemistry

Microvessel density (MVD) was detected as follows. CD31 (1:50, ab28364, Abcam) primary antibody was used for immunohistochemical staining of streptavidin peroxidase. Then the tissues were incubated at 37 °C for 30 min with secondary antibodies, developed with diaminobenzidine solution and counterstained with hematoxylin. Photographs were taken under a microscope (BX51, Olympus) in five randomly selected fields from each section, and 100 cells were counted in each area. MVD values were expressed as the number of newly formed blood vessels (CD31 positive staining cells).

### Statistical analysis

SPSS 21.0 (IBM SPSS Statistics, Chicago, IL, USA) was used for statistical analysis. The measurement data were expressed as mean ± standard deviation from at least three independent experiments. Two sets of paired data with normal distribution and homogeneity of variance were compared using the paired *t-*test, whereas unpaired data were compared using un-paired *t-*test. Data comparison among multiple groups was performed using one-way analysis of variance (ANOVA) and Tukey’s post hoc test. Cell viability at different time points was compared using two-way ANOVA while tumor volume data of different groups at different time points were compared by repeated measures ANOVA and Bonferroni post hoc test. The correlation between two indicators was analyzed by Pearson Correlation Coefficient. *p* < 0.05 indicated that the difference was statistically significant.

## Results

### miR-130b-3p is highly expressed in GC in association with poor prognosis of patients with GC

To elucidate the role of miR-130b-3p in GC and its regulatory mechanisms, we first mapped the expression box diagram of miR-130b-3p in GC in the starBase database, which showed that it was highly expressed in GC (Fig. 1a). We then examined the expression of miR-130b-3p in GC tissues using RT-qPCR, which showed significantly increased expression of miR-130b-3p in GC tissues compared with adjacent normal tissues (Fig. 1b). The expression of miR-130b-3p was closely associated with tumor size, tumor node metastasis (TNM) stage, and lymphatic metastasis of GC (Table 2). The expression of miR-130b-3p was increased in GC cells compared with the normal cell line GES-1, among which the NUGC-3 and HGC27 cell lines showed highest expression (Fig. 1c), such that they were selected for subsequent experiments. M2 macrophages have been reported to play a regulatory role in GC progression by mediating miRNAs via EVs [10, 25, 26]. To probe the relationship between M2 macrophages and miR-130b-3p, we detected the co-localization of CD206-labeled M2 macrophages by immunofluorescence and miR-130b-3p by FISH in GC tissues. This showed increased fluorescence signals and co-localization of CD206 and miR-130b-3p (Fig. 1d), thus confirming high expression of miR-130b-3p in GC.

**Fig. 1:** miR-130b-3p is highly expressed in GC. **a** The starBase database (http://www.sysu.edu.cn) predicts the expression of miR-130b in GC. The red box on the left indicates the expression of GC samples, and the purple box on the right indicates the expression of normal samples. **b** RT-qPCR was used to detect the expression of miR-130b-3p in GC tissues and adjacent normal tissues. * *p* < 0.05 vs. adjacent normal tissues. **c** RT-qPCR was used to detect the expression of miR-130b-3p in GC cells. * *p* < 0.05 vs. GES-1 cells. **d** Expression of CD206 and miR-130b-3p in GC tissues and adjacent normal tissues detected by immunofluorescence and FISH assay, respectively. Paired *t*-test was utilized for the comparison between the GC tissues and the adjacent normal tissues, and unpaired *t*-test for the comparison between other two groups

**Table 2:** Correlation between miR-130b-3p expression and clinical features of patients with GC

Character	No.	Relative miR-130b-3p expression		*p* value
		Low	High	
Gender				
Male	39	20	19	0.797
Female	24	11	13	
Age (year)				
> 50	56	27	29	0.708
≤ 50	7	4	3	
Tumor size (cm)				
> 3	44	17	27	0.014
≤ 3	19	14	5	
TNM stage				
I-II	33	9	24	0.003
III	30	22	8	
Lymphatic metastasis				
Yes	27	8	19	
No	36	23	13	0.011

*GC* gastric cancer, *miR-130b-3p* microRNA-130b-3p, *TNM* tumor node metastasis

### miR-130b-3p promotes survival, metastasis and angiogenesis of GC cells

To investigate the role of miR-130b-3p in GC cell lines, we used miR-130b-3p agomir to overexpress miR-130b-3p or miR-130b-3p antagomir to suppress its function in NUGC-3 and HGC27 GC cells. The findings of RT-qPCR suggested that miR-130b-3p agomir elevated miR-130b-3p expression, whereas miR-130b-3p antagomir reduced miR-130b-3p expression in NUGC-3 and HGC27 cells (Fig. 2a). Meanwhile, miR-130b-3p agomir promoted viability (Fig. 2b), suppressed apoptosis (Fig. 2c), enhanced migration and invasion abilities (Fig. 2d, e), increased numbers of vessel-like tubes formed in vitro (Fig. 2f), elevated Bcl-2 and VEGF expression while declining Bax and cleaved caspase3 expression (Fig. 2g, h) in NUGC-3 and HGC27 cells. The treatment with miR-130b-3p antagomir evoked opposite effects. These results indicate that downregulation of miR-130b-3p inhibits GC cell survival, metastasis, and tube formation of HUEVCs in vitro.

**Fig. 2:** Downregulation of miR-130b-3p inhibits GC cell survival, metastasis, and tube formation of HUEVCs in vitro*.***a** The expression of miR-130b-3p in cells was detected by RT-qPCR. **b** CCK-8 assay was adopted to detect the viability of cells. **c** TUNEL assay was used to detect apoptosis of cells (200 ×). **d** Transwell assay was utilized to detect the migration of cells (200 ×). **e** Transwell assay was conducted to detect the invasion of cells (200 ×). **f** Matrigel-based angiogenic assays was performed to detect numbers of vessel-like tubes formed in vitro (100 ×) **g**, **h**: Western blot assay was used to detect the expression of proteins, normalized to GAPDH in each group. * *p* < 0.05 vs. agomir-NC-transfected cells; # *p* < 0.05 vs. antagomir-NC-transfected cells. One-way ANOVA was used among multiple groups, and two-way ANOVA was performed at different time points

### miR-130b-3p promotes tumor formation and angiogenesis in GC in vivo

To investigate whether miR-130b-3p can affect GC tumor formation and angiogenesis in vivo, we injected NUGC-3 and HGC27 cells into nude mice for subcutaneous tumor formation experiments. The expression of miR-130b-3p in tumors was detected by RT-qPCR. The findings indicated that tumor bearing nude mice injected with miR-130b-3p agomir had elevated miR-130b-3p expression, whereas miR-130b-3p antagomir treatment reduced miR-130b-3p expression in NUGC-3 and HGC27 cells (Fig. 3a). There was a significant increase in tumor volume and weight (Fig. 3b, c), elevated Bcl-2 and VEGF expression, declined Bax and cleaved caspase3 expression (Fig. 3d, e), as well as increased CD31 expression (Fig. 3f) in miR-130b-3p agomir-injected nude mice. Opposite effects on these markers were seen in miR-130b-3p agomir-injected nude mice. These results indicate that miR-130b-3p promotes GC tumor formation and angiogenesis in vivo.

**Fig. 3:** miR-130b-3p induces GC tumor formation and angiogenesis in vivo*.***a** RT-qPCR was used to detect the expression of miR-130b-3p in tumors after injection of NUGC-3 and HGC27 cells. **b** Tumor volume changes in each group of nude mice. **c** Tumor weight of each group in the nude mice. **d**, **e** Western blot assay was used to detect the expression of each protein in the tumor normalized to GAPDH after injection of NUGC-3 and HGC27 cells. **f** Immunohistochemistry was used to detect CD31 expression in tumors of nude mice (200 ×). *p* < 0.05 vs. agomir-NC-injected nude mice; # *p* < 0.05 vs. antagomir-NC-injected nude mice. One-way ANOVA was used for statistical analysis among multiple groups, and repeated measure ANOVA was performed at different time points. *n* = 5 for each mouse group

### M2 macrophage-derived EVs mediate miR-130b-3p to promote survival, migration, invasion and angiogenesis of GC cells

To investigate whether the high expression of miR-130b-3p in GC is related to M2 macrophages development and their secreted EVs, we used IL-4-induced THP-1 for differentiation of M2 macrophages. Expression analysis of M2 macrophage marker genes revealed significantly higher expression of arginase and CD206 in M2 macrophages compared with THP-1 cells, suggesting that we successfully induced M2 macrophages (Fig. 4a). The expression of miR-130b-3p in NUGC-3 and HGC27 cells was significantly increased by culture with M2 macrophage culture supernatant (Fig. 4b), suggesting that miR-130b-3p is delivered to GC cells NUGC-3 and HGC27 by M2 macrophages. Further, we extracted M2 macrophage-derived EVs, which were then observed by a transmission electron microscope. EVs were solid dense bodies with a typical two-layer membrane structure, which was disc or cup-shaped. The average diameter was approximately 90 nm (Fig. 4c, d). Western blot assay was used to detect the EV marker proteins TSG101, CD63 and CD81. Compared with EVs isolated from THP-1 cells, the EV marker proteins TSG101, CD63 and CD81 were significantly increased in M2 macrophage-derived EVs (Fig. 4e), suggesting that EVs were successfully extracted from M2 macrophages, and M2 macrophages released more EVs.

**Fig. 4:** M2 macrophage-derived EVs mediate miR-130b-3p to promote survival, migration, invasion and angiogenesis of GC cells. **a** The expression of M1 and M2 macrophage marker genes was detected by RT-qPCR. **b** RT-qPCR was used to detect miR-130b-3p expression in M2 macrophages. **c** The morphology of M2 macrophage-derived EVs was observed by a transmission electron microscope (scale bar = 100 nm). **d** Nanoparticle tracking analysis of EVs size distribution. **e** Western blot analysis for the expression of EV marker proteins TSG101, CD63 and CD81 normalized to GAPDH. **f** Fluorescence staining of PKH-67-labeled M2 macrophage-derived EVs were captured by NUGC-3 and HGC27 cells and HUEVCs (400 ×). **g** The expression of miR-130b-3p in M2 macrophages was detected by RT-qPCR. **h** The CCK-8 assay was adopted to detect the viability of cells. **i** The TUNEL assay was used to detect apoptosis of cells (200 ×). **j** Transwell assay was utilized to detect the migration of cells (200 ×). **k** Transwell assay was conducted to detect the invasion of cells (200 ×). **l** Matrigel-based angiogenic assays were performed to detect numbers of vessel-like tubes formed in vitro (100 ×). **m**, **n** Western blot assay was used to detect the expression of proteins normalized to GAPDH in each group. * *p* < 0.05 vs. untreated EV group; # *p* < 0.05 vs. M2-EV + NC group. Unpaired *t* test was used for the comparison between the two groups, and two-way ANOVA was performed at different time points

To explore the uptake of EVs in GC cells, PKH67-labeled M2 macrophage-derived EVs was co-cultured with GC cells or HUEVCs for 48 h. The results showed significant green fluorescence in NUGC-3 and HGC27 cells or HUEVCs (Fig. 4f). Next, we investigated whether M2 macrophage-derived EVs promoted the function of NUGC-3 and HGC27 cells through miR-130b-3p. First, we used a lentivirus to knock down miR-130b-3p expression in M2 macrophages. RT-qPCR confirmed the reduced miR-130b-3p expression in M2 macrophages and their EVs with knockdown of miR-130b-3p (Fig. 4g). Meanwhile, compared with untreated EVs, we saw increased cell viability, migration and invasion, and decreased apoptosis of NUGC-3 and HGC27 cells (Fig. 4h-k), a significant increase in the number of tubule formation (Fig. 4l), elevated Bcl-2 and VEGF expression, and reduced Bax and cleaved caspase3 expression (Fig. 4m, n) in the M2 macrophage-derived EVs. Additional miR-130b-3p knockdown reversed the above-mentioned trends. These results together suggest that M2 macrophage-derived EVs can mediate miR-130b-3p to promote GC cell proliferation, migration, invasion, and vessel-like tube formation of HUEVCs.

### miR-130b-3p promotes proliferation, migration, invasion and angiogenesis of GC cells by inhibiting MLL3 expression

We have previously shown that the high expression of miR-130b-3p in GC cells may be related to M2 macrophage-derived EVs, and M2-macrophage-derived EVs mediated miR-130b-3p to promote GC cell proliferation, migration, invasion, and vessel-like tube formation of HUEVCs. To investigate the downstream mechanism of miR-130b-3p in GC, we predicted the downstream target genes of miR-130b-3p by microarray-based analysis. TargetScan, miRWalk, DIANA, TOOLS, StarBase, miDIP and miRDB databases, revealed 1077, 2399, 418, 50, 405 and 293 genes, respectively. Four genes identified in the intersection of the Venn maps were TBL1XR1, CLIP1, ZNF800, and MLL3 (KMT2C) (Fig. 5a). The protein-protein interaction (PPI) network of these four genes and their related genes was constructed by String, which indicated that MLL3 (KMT2C) was localized at the core (Fig. 5b, Table 3). According to the microarray-based analysis and literature review, miR-130b-3p was found to target MLL3, which is previously known to be under-expressed in GC [18]. Online website analysis showed that miR-130b-3p could target MLL3 3′-UTR. In addition, we saw that miR-130b-3p mimic significantly decreased the luciferase activity of MLL3-WT vector, but had no significant difference with the MLL3-MUT vector (Fig. 5c). The expression profile of MLL2 in GC tissues was determined by RT-qPCR, which showed that MLL3 was under-expressed in GC tissues relative to adjacent normal tissues (Fig. 5d). A negative correlation between miR-130b-3p and MLL3 in GC tissues was further revealed by Pearson correlation analysis (Fig. 5e). MLL3 expression declined in NUGC-3 and HGC27 cells with miR-130b-3p agomir treatment, while the expression elevated upon miR-130b-3p antagomir treatment (Fig. 5f). Besides, MLL3 expression was enhanced in NUGC-3 and HGC27 cells with oe-MLL3 treatment, and the reduction of MLL3 expression by miR-130b-3p agomir treatment was reversed by overexpressed MLL3 treatment (Fig. 5f). Meanwhile, decreased viability, migration and invasion, and promoted apoptosis, a decline in tubule formation, decreased Bcl-2 and VEGF expression, as well as enhanced Bax and cleaved caspase3 expression were found in NUGC-3 and HGC27 cells with oe-MLL3 treatment. The effects triggered by miR-130b-3p agomir treatment were reversed by overexpressed MLL3 treatment (Fig. 5g-m). These results suggest that miR-130b-3p targets MLL3 to promote GC cell proliferation, migration, invasion, and vessel-like tube formation of HUEVCs.

**Fig. 5:** miR-130b-3p targets MLL3 to promote GC cell proliferation, migration, invasion, and vessel-like tube formation of HUEVCs. **a** Venn plots of miR-130b’s downstream target gene results predicted by TargetScan (http://www.targetscan.org/vert_71/), miRWalk (http://mirwalk.umm.uni-heidelberg.de/), DIANA TOOLS (http://diana.imis.athena-innovation.gr/DianaTools), StarBase, miDIP (http://ophid.utoronto.ca/mirDIP/) and miRDB (http://www.mirdb.org/). **b** The PPI network diagram obtained in the String. The connection between genes indicates a relationship between genes. The color indicates the core degree. The red means the higher core degree, and the blue means lower core degree. **c** Dual luciferase reporter gene assay to detect the binding site between miR-130b-3p and MLL3. * *p* < 0.05 the mimic-NC group. **d** RT-qPCR was used to detect the expression of miR-130b-3p in GC tissues and adjacent normal tissues. * *p* < 0.05 vs. adjacent normal tissues. **e** Correlation analysis between miR-130b-3p and MLL3 by Pearson’s correlation coefficient. **f** MLL3 expression in NUGC-3 and HGC27 cells was detected by RT-qPCR. * *p* < 0.05 vs. agomir-NC-transfected cells; # *p* < 0.05 vs. antagomir-NC-transfected cells; & *p* < 0.05 vs. oe-NC-transfected cells; @ *p* < 0.05 vs. miR-130b-3p agomir + oe-NC-transfected cells. **g** CCK-8 assay was adopted to detect the viability of cells. **h** TUNEL assay was used to detect apoptosis of cells (200 ×). **i** Transwell assay was utilized to detect the migration of cells (200 ×). **j** Transwell assay was conducted to detect the invasion of cells (200 ×). **k** Matrigel-based angiogenic assays were performed to detect numbers of vessel-like tubes formed in vitro (100 ×). **l**, **m** Western blot assay was used to detect the expression of proteins normalized to GAPDH in each group. **g**-**m** * *p* < 0.05 vs. oe-NC-transfected cells; # *p* < 0.05 vs. miR-130b-3p agomir + oe-NC-transfected cells. Unpaired *t* test was used for the comparison between the two groups, and two-way ANOVA and Bonferroni test were performed for the comparison among multiple groups at different time points

**Table 3:** The core degree of genes in PPI network

Rank	Gene	Degree
1	KMT2C	6
2	TBL1XR1	5
3	ZNF800	4
4	CLIP1	1

*PPI* protein-protein interaction; Degree refers to number of interactions between genes and other genes

### MLL3 inhibits GC cell proliferation, migration, invasion, and vessel-like tube formation of HUEVCs by promoting GRHL2

Analysis of GC expression data in TCGA by GEPIA showed that MLL3 and GRHL2 had a significant positive correlation (Fig. 6a). Therefore, to study whether MLL3 involves GRHL2 in GC, we first tested the expression of GRHL2. Compared with adjacent normal tissues, GRHL2 was poorly expressed in GC tissues (Fig. 6b). The expression of GRHL2 was tightly related to tumor size, TNM stage, and lymphatic metastasis (Table 4). Relative to GES-1 cells, GRHL2 showed low expression in NUGC-3 and HGC27 cells, and overexpression of MLL3 significantly promoted GRHL2 expression (Fig. 6c). The ChIP experiment results showed an enrichment of MLL3, H3K4me1, and H3K27ac in the enhancer region of the GRHL2 gene while the enrichment increased upon overexpression of MLL3 (Fig. 6d). MLL3 and GRHL2 expression declined in NUGC-3 and HGC27 cells with sh-MLL3 treatment, while the elevated expression of GRHL2 induced by sh-MLL3 was reversed by oe-GRHL2 treatment (Fig. 6e). Meanwhile, increased cell viability, migration and invasion, and suppressed apoptosis, increased tubule formation, increased Bcl-2 and VEGF expression, but decreased Bax and cleaved caspase3 expression were found in NUGC-3 and HGC27 cells with sh-MLL3 treatment. These effects of sh-MLL3 treatment were reversed by overexpressed GRHL2 treatment (Fig. 6f-l). These results suggest that MLL3 elevates GRHL2 to restrict GC cell proliferation, migration, invasion, and vessel-like tube formation of HUEVCs.

**Fig. 6:** MLL3 elevates GRHL2 to restrict GC cell proliferation, migration, invasion, and vessel-like tube formation of HUEVCs. **a** Correlation between MLL3 and GRHL2 expression in GC obtained by GEPIA (*p* = 4.4e-16). **b** RT-qPCR was used to detect the expression of GRHL2 in GC tissues. * *p* < 0.05 vs. Adjacent normal tissues. **c** The effect of MLL3 on GRHL2 expression in NUGC-3 and HGC27 cells was detected by RT-qPCR. * *p* < 0.05 vs. GES-1 cells; # *p* < 0.05 vs. oe-NC-transfected cells (NUGC-3); & *p* < 0.05 vs. oe-NC-transfected cells (HGC27). **d** ChIP assay to detect MLL3, H3K4me1 and H3K27ac enrichment in GRHL2 gene enhancer region. * *p* < 0.05 vs. the IgG group; # *p* < 0.05 vs. the oe-NC group. **e** RT-qPCR was used to detect the expression of MLL3 and GRHL2 in each group of cells. **f** CCK-8 assay was adopted to detect the viability of cells. **g** TUNEL assay was used to detect apoptosis of cells (200 ×). **h** Transwell assay was utilized to detect the migration of cells (200 ×). **i** Transwell assay was conducted to detect the invasion of cells (200 ×). **j** Matrigel-based angiogenic assays were performed to detect numbers of vessel-like tubes formed in vitro (100 ×). **k**, **l** Western blot assay was used to detect the expression of proteins normalized to GAPDH in each group. **e**-**l** * *p* < 0.05 vs. sh-NC-transfected cells; # *p* < 0.05 vs. sh-MLL3 + oe-NC-transfected cells. Unpaired *t* test was used for the comparison between the two groups, and two-way ANOVA and Bonferroni test were performed at different time points

**Table 4:** Correlation between GRHL2 expression and clinical features of patients with GC

Character	No.	Relative GRHL2 expression		*p* value
		Low	High	
Gender				
Male	39	20	19	0.797
Female	24	11	13	
Age (year)				
> 50	56	27	29	0.708
≤ 50	7	4	3	
Tumor size (cm)				
> 3	44	27	17	0.005
≤ 3	19	4	15	
TNM stage				
I-II	33	12	21	0.045
III	30	19	11	
Lymphatic metastasis				
Yes	27	20	7	0.000
No	36	11	25	

*GRHL2* grainyhead-like 2, *GC* gastric cancer, *TNM* tumor node metastasis

### Overexpression of GRHL2 in GC cells relieves the effects of miR-130b-3p from M2 macrophage-derived EVs

To study whether the role of miR-130b-3p in M2 macrophage-derived EVs is related to changes in GRHL2 expression in GC cells, we used lentivirus to overexpress miR-130b-3p in M2 macrophages. The results suggested that miR-130b-3p expression in EVs secreted by M2 macrophages significantly improved (Fig. 7a). NUGC-3 and HGC27 cells were treated with EVs, and the expression of miR-130b-3p and GRHL2 was determined in the cells. The results showed increased miR-130b-3p and reduced GRHL2 expression in NUGC-3 and HGC27 cells with M2 macrophage-derived EVs and oe-miR-130b-3p treatment, while GRHL2 expression was elevated in cells upon treatment with M2 macrophage-derived EVs, oe-miR-130b-3p and oe-GRHL2 (Fig. 7b). Meanwhile, greater cell viability, migration and invasion, and suppressed apoptosis of MGC803 and SGC790 cells, an enhanced tubule formation, increased Bcl-2 and VEGF expression, along with reduced Bax and cleaved caspase3 expression were found in NUGC-3 and HGC27 cells treated with M2 macrophage-derived EVs and oe-miR-130b-3p. The trend was reversed by supplement of the overexpressed GRHL2 treatment (Fig. 7c-i). These results suggest that MLL3 elevates GRHL2 to restrict GC cell proliferation, migration, invasion, and vessel-like tube formation of HUEVCs, and that overexpression of GRHL2 in GC cells can alleviate the effects of miR-130b-3p from M2 macrophage-derived EVs.

**Fig. 7:** Overexpression of GRHL2 in GC cells alleviates the effects of miR-130b-3p from M2 macrophage-derived EVs. **a** RT-qPCR detection of miR-130b-3p expression in M2 macrophage-derived EVs. * *p* < 0.05 vs. cells with M2-EV + oe-NC treatment. **b** RT-qPCR detection of miR-130b-3p and GRHL2 expression in NUGC-3 and HGC27 cells treated with EVs. **c** CCK-8 assay was adopted to detect the viability of cells. **d** TUNEL assay was used to detect apoptosis of cells (200 ×). **e** Transwell assay was utilized to detect the migration of cells (200 ×). **f** Transwell assay was conducted to detect the invasion of cells (200 ×). **g** Matrigel-based angiogenic assays were performed to detect numbers of vessel-like tubes formed in vitro (100 ×). **h**, **i** Western blot assay was used to detect the expression of proteins normalized to GAPDH in each group. **b**-**i** * *p* < 0.05 vs. cells with M2-EV + oe-NC treatment; # *p* < 0.05 vs. cells with M2-EV + oe-miR-130b-3p treatment. One-way ANOVA and Tukey’s test were used for the comparison among multiple groups, and two-way ANOVA and Bonferroni test were performed at different time points

### Knockdown of miR-130b-3p in M2 macrophage-derived EVs or overexpression of GRHL2 in GC cells inhibits tumor growth and angiogenesis

To study whether miR-130b-3p from EVs or overexpression of GRHL2 in GC cells could affect tumor growth in vivo, we performed tumor xenograft studies in nude mice. We directly overexpressed GRHL2 in NUGC-3 and HGC27 cells or by using lentivirus to knockdown miR-130b-3p in M2 macrophages and extracted EVs into nude mice. Tumor tissue samples were collected 4 weeks later for the detection of relevant indicators. Reduced miR-130b-3p and increased GRHL2 expressions were found in mice injected with M2 macrophage-derived EVs + miR-130b-3p knockdown, whereas the expression of miR-130b-3p did not significantly change in mice injected with oe-GRHL2, with increased GRHL2 expression (Fig. 8a). Significant reduction in tumor volume and weight, decreased Bcl-2 and VEGF expression, elevated Bax and cleaved caspase3 expression, as well as declined CD31 were found in nude mice injected with M2 macrophage-derived EVs + miR-130b-3p knockdown or oe-GRHL2 (Fig. 8b-f). These results indicate that knockdown of miR-130b-3p in M2 macrophage-derived EVs or overexpression of GRHL2 inhibits GC tumor formation and angiogenesis in vivo.

**Fig. 8:** Knockdown of miR-130b-3p in M2 macrophage-derived EVs or overexpression of GRHL2 inhibits GC tumor growth and angiogenesis in vivo. **a** RT-qPCR detection of miR-130b-3p and GRHL2 expression in tumors after injection of NUGC-3 and HGC27 cells. **b** Tumor volume change in each group. **c** Tumor weight change in each group. **d**, **e** Western blot analysis to detect the expression of each protein in tumor tissues normalized to GAPDH after injection of NUGC-3 and HGC27 cells. **f** CD31 expression in each group of tumors (200 ×). * *p* < 0.05 vs. mice without treatment; # *p* < 0.05 vs. mice injected with M2-EV-NC; & *p* < 0.05 vs. mice injected with oe-NC. One-way ANOVA and Tukey’s test were used for the comparison among multiple groups, and two-way ANOVA and Bonferroni test were performed at different time points. *n* = 5 for each mouse group

## Discussion

Interestingly, the miRNA transfer by EVs results in the development of chemoresistance in many tumor types [27]. Upregulation or downregulation of several miRNAs has been found in multiple cancer types, including GC, digesting that miRNA profiling might be a new biomarker for diagnosis, prognosis prediction, and assessment of treatment response [28, 29]. It is known that M2 macrophages can regulate GC progression by EV-mediated miRNA [10, 25, 26]. In this present study, we aimed to investigate the mechanism of miR-130b-3p in M2 macrophage-derived EVs during the development of GC through regulation of MLL3 and GRHL2. Collectively, our results suggest that miR-130b-3p in M2 macrophage-derived EVs contributes to the development of GC through regulation of MLL3 and GRHL2.

We found that miR-130b-3p was highly expressed in GC and that its expression was related to GC patients’ survival. In addition, we also found that miR-130b-3p promoted survival, metastasis and angiogenesis of GC cells as well tumor growth and angiogenesis in vivo. A prior study has yielded similar results demonstrating that miR-130b expression was elevated in GC tissues relative to matched normal tissues, and that the upregulated miR-130b promoted cell viability and reduced death of GC cells [30]. Another study likewise showed increased miR-130b-5p expression in GC cell lines, and that GC cells with overexpressed miR-130b-5p had potentiated cell proliferation, colony formation, as well as migratory and invasive capacities [31]. High expression of other miRNAs, such as miR-130, has been observed in advanced GC tissues, which was similarly associated with risk for distant metastasis, lymph node metastasis, and poor long-term survival [28].

Additionally, results of this study suggested that M2 macrophage-derived EVs mediated delivery of miR-130b-3p to promote survival, migration, invasion and angiogenesis of GC cells. A recent study has elucidated that M2 macrophages-derived miR-328-containing EVs are able to stimulate pulmonary fibrosis in a rat model through silencing FAM13A [32]. Meanwhile, another article has provided evidence that EV-enclosed miR-21 derived from tumor-associated macrophages constitute a promising adjunct treatment approach for patients with GC, particularly those with cisplatin-resistant GC [25]. The contribution of tumor-associated M2 macrophages to the progression and development of GC has already been reported [33, 34]. Likewise, M2 macrophage polarization induced by exposure to mesenchymal stromal cells derived from GC cells facilitates the metastasis and epithelial-mesenchymal transition, while M2 macrophage differentiation triggered by IL-6 potentiates proliferation and migration capabilities of GC cells [35, 36]. Moreover, transfer of M2 macrophage-derived EVs to colon cancer cells could explain the manner in which immune cells are implicated in tumor progression [37]. Until now, the association between EVs and miR-130b-3p has seldom discussed, and this topic needs further verification.

Another important finding of our study was that miR-130b-3p promoted proliferation, migration, invasion and angiogenesis of GC cells by inhibiting MLL3 and GRHL2. An earlier study has shown that MLL3 is under-expressed in GC and plays a vital role in GC development [18]. Another study reported that GC susceptibility has a close association with the S3660L mutation of MLL3 gene [17]. H3K27 acetyltransferases (CBP/p300) and histone H3K4me1/2 methyltransferases (MLL3/MLL4) are the main epigenomic enhancers [38]. The transcription factor GRHL2, which inhibits oncogenic epithelial-mesenchymal transition in breast cancer, is silenced in MLL3-knockout cells [21]. Xiang et al. found that GRHL2 overexpression suppressed the ability of invasion and migration of GC cells, and that GRHL2 reduced the expression of matrix metalloproteinases [39]. Another study has revealed that exogenous GRHL2 transfected into GC SGC7901 cells contributed to the suppressed proliferation and promoted apoptosis, as well as decreased c-Myc and Bcl-2 expression in culture [40]. Furthermore, the present in vivo experiment suggesting that knockdown of miR-130b-3p in M2 macrophage-derived EVs or overexpression of GRHL2 in GC cells inhibited tumor growth and angiogenesis is in accord with the corresponding in vitro results.

## Conclusion

In conclusion, this study highlights that miR-130b-3p in M2 macrophage-derived EVs contributes to the development of GC through regulating MLL3 and GRHL2 (Fig. 9). Moreover, EVs have a potential capability for prognostic prediction for patients with GC. Despite the growing focus on the role of EVs in GC, there are still challenges to be addressed before EVs can be applied in the clinical treatment of GC.

**Fig. 9:** miR-130b-3p from M2 macrophage-derived EVs regulates the expression of GRHL2 by MLL3, thereby participating in GC progression. In GC, miR-130b-3p from M2 macrophage-derived EVs can target MLL3 expression. The downregulation of MLL3 promotes the reduction of H3K4me1 and H3K27ac enrichment in the GRHL2 enhancer, thereby inhibiting the expression of GRHL2, and ultimately promoting the survival of GC cells

## Data Availability

The datasets generated/analysed during the current study are available.

## Abbreviations

miRNAs: microRNAs
EVs: Extracellular vesicles
GC: Gastric cancer
MLL3: Mixed lineage leukemia 3
GRHL2: Grainyhead-like 2
HUEVCs: Human umbilical endothelial vein cells
IL-4: Interleukin-4
FISH: Fluorescence in situ hybridization
DIG: Double-digoxigenin
TSA: Tyramide Signal Amplification
DAPI: 4′, 6-diamidino-2-phenylindole
NCs: Negative controls
TSG101: Tumor susceptibility gene 101
RT-qPCR: Reverse transcription quantitative polymerase chain reaction
GAPDH: Glyceraldehyde phosphate dehydrogenase
Bax: B-cell lymphoma-2 (Bcl-2) associated protein X
IgG: Immunoglobulin G
WT: Wild-type
MUT: Mutant type
3′-UTR: 3′-untranslated region
ChIP: Chromatin immunoprecipitation
CCK-8: Cell counting kit-8
TUNEL: Terminal dexynucleotidyl transferase (TdT)-mediated 2′-deoxyuridine 5′-triphosphate (dUTP) nick end labeling
MVD: Microvessel density
ANOVA: Analysis of variance
TNM: Tumor node metastasis
PPI: Protein-protein interaction
